The article "Long non-coding RNA ROR1-AS1 induces tumorigenesis of colorectal cancer by affecting Wnt/β-catenin signaling pathway" was retracted in 2020. Reasons: duplicated images; signs of a paper mill; concerns about the data.

# Long non-coding RNA ROR1-AS1 induces tumorigenesis of colorectal cancer by affecting Wnt/β-catenin signaling pathway

**DOI:** 10.1042/BSR20191453

**Published:** 2019-11-22

**Authors:** Wei Wang, Weihong Zheng, Lei Zhang, Ke Li

**Affiliations:** 1 Department of General Surgery, Zhejiang Chinese Medicine and Western Medicine Integrated Hospital/Hangzhou Red Cross Hospital, 208 East Huancheng Road, Hangzhou Zhejiang, China; 2 School of Life Science, Huzhou University, 759 Erhuan East Road, Huzhou, Zhejiang, China; 3 Department of Anorectal Surgery, the Second Affiliated Hospital of Zhejiang Chinese Medical University, 318 Chaowang Road, Hangzhou, Zhejiang, China

**Keywords:** colorectal cancer, Long noncoding RNA, ROR1-AS1, Wnt/β-catenin signaling pathway

## Abstract

Recent studies have discovered that long noncoding RNAs (lncRNAs) play an important role in malignant tumors. In this research, lncRNA ROR1-AS1 was selected to identify how it affects the development of colorectal cancer (CRC). ROR1-AS1 expression was detected by RT-qPCR in CRC tissue samples. ROR1-AS1 expression level and patients’ overall survival time were analyzed. Functional experiments were conducted to identify the changes of biological behaviors in CRC cells after knockdown of ROR1-AS1. Moreover, we also explored the underlying mechanism. Detection of ROR1-AS1 expression level in patients’ tissues showed that ROR1-AS1 was higher in CRC tissues than that in adjacent ones. ROR1-AS1 expression was negatively associated with patients’ overall survival time. Cell growth ability was inhibited due to knockdown of ROR1-AS1 *in vitro*. Moreover, cell migration and invasion were repressed after ROR1-AS1 knockdown. Furthermore, due to knockdown of ROR1-AS1, the targeted proteins in Wnt/β-catenin signaling pathway were suppressed. These results suggest that ROR1-AS1 could enhance cell metastasis and proliferation via inducing Wnt/β-catenin signaling pathway, which might offer a potential therapeutic target in CRC.

## Introduction

The incidence rate of colorectal cancer (CRC) remains high both in males and females worldwide [1–3]. A total of 1.36 million CRC cases were diagnosed annually globally and almost 0.6 million cases died of CRC [2]. Although the technological advances have been made in early detection and intervention for the past decades, the prognosis of patients with CRC is still dismal, with poor 5-year survival rate [4]. Thus, it is crucial to uncover the molecular mechanism underlying the progression of CRC and find out potential targets to improve the poor prognosis of this malignant tumor.

As one subtype of noncoding RNA (ncRNA), long ncRNAs (lncRNAs) regulate a variety of cellular processes and pathways in the development of many diseases [5]. For example, LncRNA NEAT1 is highly expressed and participates in development of Huntington’s disease [6]. LncRNA HOTAIR facilitates the development of Parkinson’s disease through LRRK2 [7]. Recent studies also demonstrate that ncRNA also participates in progression of cancers. For instance, down-regulation of lncRNA linc-ITGB1 inhibits cell invasion, cell migration and epithelial–mesenchymal transition in non-small cell lung cancer by decreasing Snail expression [8]. Expression level of lncRNA-CCHE1 is positively related to the malignancy of colorectal carcinoma and it regulates ERK/COX-2 pathway [9]. Through regulating the stability of DNMT1 and depressing the expression of tumor suppressors, lncRNA LUCAT1 promotes esophageal squamous cell carcinoma formation and cell metastasis [10]. Activated by ZEB1, lncRNA HCCL5 accelerates cell viability, cell migration, epithelial–mesenchymal transition and the malignancy of hepatocellular carcinoma [11]. LncRNA SChLAP1 contributes to the development of aggressive prostate cancer by antagonizing the function of the SWI/SNF complex [12]. However, how lncRNA ROR1-AS1 participates in the progression of CRC remains unknown.

In the present study, ROR1-AS1 was remarkably higher expressed in CRC tissues when compared with adjacent normal tissues. Moreover, ROR1-AS1 promoted the proliferation and invasion of CRC *in vitro*. Our further experiments also showed that ROR1-AS1 participated in tumorigenesis of CRC through Wnt/β-catenin signaling pathway.

## Materials and methods

### Clinical samples

Tumor samples and the adjacent tissues (≥5 cm away from the edge of tumor) were gathered from CRC patients (*n*=52) who underwent surgery at Zhejiang Chinese Medicine and Western Medicine Integrated Hospital/Hangzhou Red Cross Hospital between 2014 and 2017. Written informed consent was taken before operation. All fresh tissues were preserved at −80°C. The present study was approved as the Human Research Ethics Committee from Zhejiang Chinese Medicine and Western Medicine Integrated Hospital/Hangzhou Red Cross Hospital required.

### Cell culture

The American Type Culture Collection (ATCC) offered human CRC cell lines HCT116, HT29, SW620, SW480 and normal human colonic epithelial cells (NCM460), which were then cultured in Roswell Park Institute Memorial 1640 (RPIM-1640) supplemented with 5% fetal bovine serum (FBS) in an incubator containing 5% CO_2_ at 37°C.

### Cell transfection

We purchased short hairpin RNA (shRNA) targeting ROR1-AS1 (sh-ROR1-AS1), scrambled oligonucleotides (NC) from GenePharma (Shanghai, China). The complementary DNA encoding ROR1-AS1 was PCR-amplified, which was then inserted into pcDNA3.1 (Invitrogen). Those treated cells were used for following experiments.

### RNA extraction and RT-qPCR

Twenty-four hours after transfection, total RNA was extracted from CRC cells or tumor tissues from CRC patients using TRIzol reagent (Invitrogen; Thermo Fisher Scientific, Inc.). First-strand cDNA was synthesized using the Transcriptor first strand cDNA synthesis kit (Takara Biotechnology Co., Ltd., Dalian, China) according to the manufacturer’s instructions. Following are the primers used for RT–qPCR: ROR1-AS1 primers forward 5′- CTGACGAAACACTGGAACTC-3′, reverse 5′-GTCTGATTTGGTAGCTTGGATG-3′; GAPDH primers forward 5′-CCAAAATCAGATGGGGCAATGCTGG-3′ and reverse 5′-TGATGGCATGGACTGTGGTCATTCA-3′. Thermal cycle was as follows: 30 s at 95°C, 5 s for 40 cycles at 95°C, 35 s at 60°C.

### MTT assay

Before transfection, CRC cells (1000 cells/well) were seeded into 96-well plate for 12 h. After they were cultured at different times (0, 24, 48, and 72 h), 15 μl MTT was added to each well and incubated for 4 h. To stop the reaction, they were added with 100 μl dimethyl sulfoxide. Absorbance at 490 nm was assessed using an ELISA reader system (Multiskan Ascent, LabSystems).

### Colony formation assay

Those transfected cells were placed in a six-well plate for 2 weeks. Cell colonies were treated with methanol for 30 min. Then 0.5% Crystal Violet was used for staining for 5 min. Colonies containing more than 50 cells were counted and the mean colony numbers were calculated. Analysis was conducted with Image-Pro Plus 6.0.

### Wound healing assay

Cells, seeded in six-well plates, were incubated overnight. After scratching with a pipette tip, cells were cultured in serum-free DMEM. Relative distance was viewed under a light microscope (Olympus Corp.) at 48 h. Each assay was independently repeated in triplicate.

### Transwell assay

A total of 2 × 10^4^ cells in serum-free DMEM were replanted in the upper chamber which was coated with 30 μl of Matrigel (BD Biosciences, San Jose, CA, U.S.A.). DMEM and FBS were added into the bottom chamber. After 24 h of incubation, the cells were immersed with 4% paraformaldehyde for 10 min and stained with 1% Crystal Violet for 30 min to remove any uninfected cells from the upper chamber. Next, cells were counted and photographed in randomly selected fields with a Leica DMI4000B microscope (Leica Microsystems, Heidelberg, Germany).

### Western blot analysis

Cell samples were washed with precooled PBS and then lysed with cell lysis solution (RIPA). Protein concentration was detected using BCA (Thermo Fisher Scientific Inc., MA, U.S.A.). The proteins were transferred on to a PVDF membrane, blocked in TBST (25 mM Tris, 140 mM NaCl and 0.1% Tween 20, pH 7.5) containing 5% skimmed milk and incubated for 2 h. The proteins were incubated with the primary antibody of target proteins including Wnt3a, β-catenin, C-myc and Survivin (Abcam Inc., Cambridge, MA, U.S.A.) in Wnt/β-catenin signaling pathway and GAPDH (Abcam Inc., Cambridge, MA, U.S.A.) and incubated at 4°C overnight. After being washed (3 × 10 min) with TBST, the secondary antibody was added and incubated at room temperature for 1 h. The results were analyzed by ImageJ software.

### Statistical analysis

GraphPad Prism 5.0 was adopted to conduct the statistical analysis. Data were expressed as mean ± SD. Student’s *t* test and Kaplan–Meier method were utilized. It was considered to be of statistical significance, when *P*-value was less than 0.05.

## Results

### ROR1-AS1 expression level in CRC tissues

RT-qPCR was conducted for detecting ROR1-AS1 expression in 52 patients’ tissues. ROR1-AS1 was significantly up-regulated in CRC tissue samples (Figure 1A). ROR1-AS1 expression level was higher in CRC cells than that in NCM460 (Figure 1B and Figure S1).

**Figure 1:** Expression levels of ROR1-AS1 were increased in CRC patients (**A**) ROR1-AS1 expression was significantly increased in the CRC tissues compared with adjacent tissues. (**B**) Expression levels of ROR1-AS1 were determined in the human CRC cell lines and NCM460 by RT-qPCR. *P<0.05.

### The association between ROR1-AS1 expression level and the prognosis of CRC patients

We divided 52 patients into two groups, high ROR1-AS1 level and low ROR1-AS1 level, via median expression. Kaplan–Meier analysis showed that patients in high ROR1-AS1 level group had a poorer overall survival compared with those in low ROR1-AS1 level group (Figure 2).

**Figure 2:** The association between ROR1-AS1 expression level and the prognosis of CRC patients Expression levels of ROR1-AS1 were negatively associated with patients’ overall survival time. *P<0.05.

### Cell proliferation was inhibited in CRC cells via knockdown of ROR1-AS1

As ROR1-AS1 expression level was the highest in SW620 among four CRC cell lines, SW620 cells were used for the transfection of ROR1-AS1 shRNA or scrambled oligonucleotides (NC). Then RT–qPCR was utilized for detecting the ROR1-AS1 expression (Figure 3A). Moreover, results of MTT assay revealed that the cell growth ability of CRC cells was obviously repressed via knockdown of ROR1-AS1 (Figure 3B). The outcome of colony formation assay also revealed that the number of colonies was remarkably reduced via knockdown of ROR1-AS1 in CRC cells (Figure 3C).

**Figure 3:** ROR1-AS1 promoted CRC cell proliferation and metastasis (**A**) ROR1-AS1 expression in CRC cells transfected with ROR1-AS1 shRNA (sh-ROR1-AS1) or scrambled oligonucleotides (NC) was detected by RT-qPCR. GAPDH was used as an internal control. (**B**) MTT assay revealed that the cell growth ability of CRC cells was obviously repressed in sh-ROR1-AS1 group compared with NC group. (**C**) Colony formation assay also revealed that the number of CRC cell colonies was remarkably reduced in sh-ROR1-AS1 group compared with NC group. (**D**) The migrated ability of CRC cells was significantly decreased in sh-ROR1-AS1 group compared with NC group (magnification: 40×). (**E**) Transwell assay showed that number of invaded CRC cells was significantly decreased in sh-ROR1-AS1 group compared with NC group (magnification: 40×). The results represent the average of three independent experiments (mean ± standard error of the mean). *P<0.05.

### Cell migration and invasion was inhibited in CRC cells via knockdown of ROR1-AS1

Wound healing assay results revealed that the relative migrated ability of SW620 CRC cells was obviously repressed via knockdown of ROR1-AS1 (Figure 3D). The outcome of Transwell assay also revealed that the number of invaded cells was remarkably reduced via knockdown of ROR1-AS1 in SW620 CRC cells (Figure 3E).

### The interaction between Wnt/β-catenin signaling pathway and ROR1-AS1 in CRC

To explore the underlying mechanism of ROR1-AS1 function in CRC, RT-qPCR and Western blot assay were conducted to detect the target proteins in Wnt/β-catenin signaling pathway such as Wnt3a, β-catenin, C-myc and Survivin in SW620 CRC cells. RT-qPCR results showed that Wnt3a, β-catenin, C-myc and Survivin could be down-regulated via knockdown of ROR1-AS1 (Figure 4A). Western blot assay results showed that Wnt3a, β-catenin, C-myc and Survivin could be down-regulated via knockdown of ROR1-AS1 (Figure 4B). These results suggested that ROR1-AS1 participated in regulation of Wnt/β-catenin signaling pathway and further promoted CRC development and metastasis.

**Figure 4:** ROR1-AS1 promoted CRC tumorigenesis and activated Wnt/β-catenin signaling pathway (**A**) RT-qPCR results revealed that the expression of target proteins in Wnt/β-catenin signaling pathway was down-regulated in sh-ROR1-AS1 group compared with NC group. (**B**) Western blot assay results revealed that the expression of target proteins in Wnt/β-catenin signaling pathway was down-regulated in sh-ROR1-AS1 group compared with NC group. The results represent the average of three independent experiments (mean ± standard error of the mean). *P<0.05.

## Discussion

Numerous studies have proved that ncRNAs take part in a variety of important biological processes, including tumor growth. Previously, evidence have revealed that several lncRNAs participate in the development of CRC. For instance, lncRNA TP73AS1 promotes cell apoptosis of CRC by sponging miR103 [13]. LncRNA RUNX1-IT1 acts as a tumor suppressor in CRC by inhibition of cell migration and cell proliferation, which suggests RUNX1-IT1 could function as a novel diagnostic biomarker [14]. In addition, lncRNA H19 promotes 5-Fu resistance in CRC via sponging to miR-194-5p [15].

Located in 1p31.3, ROR1-AS1 is a newly discovered lncRNA which is first discovered in mantle cell lymphoma [16]. In the current study, we conducted experiments to identify the role of ROR1-AS1 in CRC. Results showed that ROR1-AS1 was up-regulated in CRC samples and was associated with patients’ prognosis. Besides, CRC proliferation and invasion were found to be inhibited via knockdown of ROR1-AS1. Above results indicated that ROR1-AS1 promotes tumorigenesis of CRC and might act as an oncogene.

Previous researches have suggested that aberrant activation of the Wnt/β-catenin signaling pathway plays an important role in regulating development of several human cancers. For instance, Wnt/β-catenin signaling pathway was activated by WDR34 in hepatocellular carcinoma [17]. SPINK5 modulates Wnt/β-catenin signaling pathway in esophageal cancer [18]. Wnt/β-Catenin/Axin2 signaling activated by c-Myb promotes proliferation and metastasis of breast cancer [19]. Wnt10a acts as an oncogene in CRC through activating Wnt/β-catenin signaling [20]. As Wnt3a, β-catenin, C-myc and Survivin were the target proteins in Wnt/β-catenin signaling pathway, we detected the expression of those proteins in CRC cells after knockdown of ROR1-AS1. Results showed that target proteins in Wnt/β-catenin signaling pathway could be down-regulated via knockdown of ROR1-AS1. All the results above suggested that ROR1-AS1 might promote tumorigenesis of CRC via activating Wnt/β-catenin signaling pathway.

## Conclusion

Above data identified that ROR1-AS1 could enhance CRC cell proliferation and invasion through activating Wnt/β-catenin signaling pathway. These findings indicate that ROR1-AS1 may contribute to therapy for CRC as a candidate target.

## Abbreviations

CRC: colorectal cancer
FBS: fetal bovine serum
lncRNA: long noncoding RNA
NCM460: normal human colonic epithelial cell
ncRNA: noncoding RNA
shRNA: short hairpin RNA
